# Screening of Key Prognosis Genes of Lung Adenocarcinoma Based on Expression Analysis on TCGA Database

This article has been retracted.

**DOI:** 10.1155/2022/4435092

**Published:** 2022-12-26

**Authors:** Youfeng Shen, Xiaoqing Tang, Xiaoqin Zhou, Yuanxue Yi, Yuan Qiu, Jian Xu, Xingzhong Tian

**Affiliations:** ^1^Chongqing Precision Medical Industry Technology Research Institute, Chongqing 400000, China; ^2^Department of Laboratory Medicine, Nanan People's Hospital, Chongqing 400060, China; ^3^Department of Laboratory Medicine, Kaizhou District People's Hospital, Chongqing 405400, China; ^4^College of Laboratory Medicine, Chongqing Medical University, Chongqing 400000, China; ^5^The Fifth Hospital of Zhangjiakou, China

## Abstract

**Objective:**

The data of lung adenocarcinoma- (LUAD-) related gene expression profiles were mined from the Cancer Genome Atlas (TCGA) database using bioinformatics methods and potential biomarkers related to the occurrence, development, and prognosis of LUAD were screened out to explore the key prognostic genes and clinical significance.

**Methods:**

Following the LUAD gene expression profile data that were initially exported from the TCGA database, R software DESeq2 was employed to analyze the difference between the expression profiles of LUAD and normal tissues. The R package “clusterProfiler” was subsequently utilized to perform gene ontology (GO) and Kyoto Encyclopedia of Genes and Genomes (KEGG) pathway analyses of the differential genes. A protein-protein interaction (PPI) network was constructed via the String database, and cytohubba, a plugin of Cytoscape, was applied to screen hub genes using the MCC algorithm. The Gene Expression Profile Data Interactive Analysis (GEPIA) was used to analyze expressions of 10 candidate genes in LUAD samples and healthy lung samples, and the selected genes were employed for survival analysis.

**Results:**

A total of 1,598 differential genes were identified through differential analyses and data mining, with 1,394 genes upregulated and 204 downregulated. A total of 10 hub genes CCNA2, CDC20, CCNB2, KIF11, TOP2A, BUB1, BUB1B, CENPF, TPX2, and KIF2C were obtained using the cytohubba plugin. The results of the GEPIA analysis indicated that compared with normal lung tissue, the mRNA expression level of the described hub genes in LUAD tissue was significantly increased (*P* < 0.05). Survival analysis revealed that these genes had a significant impact on the overall survival time of LUAD patients (*P* < 0.05).

**Conclusion:**

The previously described key genes related to LUAD identified in the TCGA database may be used as potential prognostic biomarkers, which will contribute to further comprehension of the occurrence and development of LUAD and provide references for its diagnosis and treatment.

## 1. Introduction

Lung cancer has become the most common malignant tumor worldwide and the leading cause of cancer-related death, which is usually closely associated with a poor prognosis. According to the latest report of the Global Cancer Statistics Center, lung cancer has the highest incidence and mortality among all male patients with malignant tumors, while the incidence of lung cancer in female patients is lower than that of breast cancer and colon cancer, and the mortality rate is second only to that of breast cancer [1]. Lung adenocarcinoma (LUAD) is the most common pathological type of non-small-cell lung cancer, accounting for 85% of the incidence of lung cancer [2, 3]. In recent years, it has been characterized by rapid onset, younger age, high mortality, and poor prognosis. Therefore, it is increasingly important to explore new prognostic genes for LUAD in the era of precision medicine.

The Cancer Genome Atlas (TCGA) is currently the largest tumor gene expression profile database in the world, including clinical sample data and genomic data of a variety of tumors, which promotes the discovery of de novo markers [4]. Based on TCGA studies, it was found that ZNF695 may be indirectly associated with proliferation in lung cancer. In LUAD, ZNF695 expression was significantly higher in bronchial and magnolia mRNA isoforms, exhibiting overrepresentation of growth and proliferation pathways, respectively [5]. RRM2 is upregulated in LUAD, and high RRM2 expression is associated with clinical progression and is considered an independent risk factor for OS in LUAD patients [6].

In this study, based on the TCGA database, the bioinformatics method was applied to screen and integrate the expression profile data of LUAD, analyze and find differential genes, and perform functional enrichment analysis, PPI network construction, key gene screening, survival analysis, etc. This provides a theoretical basis for further screening of prognostic genes in LUAD.

## 2. Material and Methods

### 2.1. Data Acquisition

“Lung cancer” was used as the keyword to search in TCGA (https://portal.gdc.cancer.gov/) database, and the data category was selected as “transcriptome profiling”. Publicly available genomic data on LUAD were downloaded, including 551 samples, of which 497 were LUAD-associated and 54 were normal samples. The clinical information of 486 cases including gender, survival status, survival time, race, and pathological stage were obtained for subsequent analysis.

### 2.2. Method

#### 2.2.1. Data Processing and Screening of Differentially Expressed Genes

After removing the repeated genes in the downloaded original data and the genes with 0 expressions in the multiple copies, differential analysis and screening of differentially expressed genes were undertaken using the R software package DESeq2. The selection criteria are as follows: |log2(FoldChange)| > 3 and correct after *P* values (false discovery rate, FDR) <0.05. The top 50 cluster heat map of differential genes between normal samples and tumor samples was drawn using the R software package PheATMap. The R package GGPubR and GGThemes were used to draw the volcano map to observe the relationship between differential change times and FDR.

#### 2.2.2. GO and KEGG Enrichment Analysis of Differential Genes

Based on the R4.1.1 environment, four R packages (clusterProfiler, Stringr, org.hs.eg.db, and ggploT2) were performed using gene function analysis, including Biological process (BP), Cellular components (CC) and Molecular function (MF), and pathway analysis based on KEGG. The screening criterion is as follows: FDR < 0.05. The top 10 results of significantly enriched BP, CC, MF, and KEGG pathways were selected and graphed.

#### 2.2.3. Protein Interaction Network Construction and Hub Gene Screening

The STRING Database (https://string-db.org/) is an online analytical tool for identifying known proteins or predicting protein-protein interactions. The selected differential genes were imported into the database for protein-protein interaction (PPI) analysis, and the confidence score threshold was set to 0.9. The PPI network results were then imported into Cytoscape 3.6.1 in TSV format for visualization. The top 10 genes were screened from the PPI network as hub genes using the MCC method in the Cytohubba plugin of Cytoscape.

#### 2.2.4. Expression of 10 Hub Genes in LUAD

Using GEPIA (http://gepia.cancer-pku.cn/index.html) online analysis website (“Datasets” select “LUAD”, “Matched normal data” select “TCGA normal and the Genotype-Tissue Expression (GTEx) data”), the expression of 10 candidate genes in LUAD tumor samples and normal lung samples were analyzed and compared.

#### 2.2.5. Survival Analysis of Key Genes

Based on R 4.1.1 environment, Survival package and SurvMiner package were used for survival analysis, Kaplan-Meier survival curve construction, and to estimate and screen the prognostic markers. The log-rank test was used to evaluate the survival difference between the expression level of key genes and the overall survival rate of lung adenocarcinoma patients, and *P* < 0.05 was considered statistically significant.

## 3. Result

### 3.1. Screening of Differentially Expressed Genes in LUAD

In this study, a total of 551 LUAD-related patient data were downloaded, collated, and analyzed from the TCGA database, including 497 tumor samples and 54 normal samples. DESeq2 R package was used for differential analysis, and a total of 1598 differential genes were screened, including 1397 upregulated genes and 204 downregulated genes. A heat map of the top 50 genes with the most significant differences (Figure 1(a)) and a volcano plot of the 1,598 differential genes (Figure 1(b)) were plotted.

### 3.2. Functional Enrichment Analysis of Differential Genes

R software was used for GO and KEGG enrichment analysis of 1,394 upregulated genes and 204 downregulated genes, respectively. The GO results of 1,394 upregulated genes showed that they were mainly involved in the positive regulation of RNA polymerase II transcription, mitotic mitosis, nucleosome assembly, and other biological processes, but they were also involved in the extracellular region, extracellular space, protein extracellular matrix, nucleosome, and other cytological components. It also plays the molecular biological functions of serine endothase activity, calcium ion binding, nucleosome binding, chromatin binding, and so on (Figure 2(a)). KEGG enrichment results showed that the pathways involved mainly protein digestion and absorption, tumor transcription dysregulation, and amino acid biosynthesis, etc. (Figure 2(b)). The 204 downregulated genes were mainly involved in biological processes such as oxygen transport, synaptic transmission, and cell response to TGF-*β* stimulation. It also participates in cytological components such as hemoglobin-haptoglobin complex, lateral basement plasma membrane, extracellular space, and cell-cell junction. It also plays molecular biological functions such as oxygen transporter activity, haptoglobin binding, iron binding, peroxidase activity, and G-protein-coupled acetylcholine receptor activity (Figure 2(c)). KEGG enrichment results also showed that the pathways involved mainly neural ligand-receptor interaction, calcium signaling pathway, PI3K-Akt signaling pathway, etc. (Figure 2(d)).

### 3.3. Protein Interaction Network Construction and Central Gene Screening

A PPI interaction network was constructed for LUAD-related differentially expressed genes based on String database. The MCC algorithm in Cytoscape plug-in CytoHubba was used to screen the top 50 genes in the PPI network to construct the protein interaction network diagram (Figure 3(a)). The top 10 genes were selected as central genes, which were *CCNA2*, *CDC20*, *CCNB2*, *KIF11*, *TOP2A*, *BUB1*, *BUB1B*, *CENPF*, *TPX2*, and *KIF2C* (Figure 3(b).

### 3.4. GEPIA Analysis of the Expression of 10 Hub Genes in Lung Adenocarcinoma

Compared with normal lung tissue, the mRNA expression levels of 10 hub genes (*CCNA2*, *CDC20*, *CCNB2*, *KIF11*, *TOP2A*, *BUB1*, *BUB1B*, *CENPF*, *TPX2*, and *KIF2C*) in LUAD tissues were significantly increased (*P* < 0.05, Figure 4).

### 3.5. Survival Analysis of Key Genes

The survival of 10 hub genes screened from PPI network was analyzed using R software, and the Kaplan-Meier survival curve was drawn. Log-rank test revealed that these genes had a significant effect on the overall survival of patients with LUAD (*P* < 0.05, Figure 5). Therefore, it can be concluded that these genes play an important role in the occurrence and development of LUAD.

## 4. Discussion

Based on the TCGA database, this study used bioinformatics methods to explore the key genes related to the development and prognosis of LUAD. A total of 551 LUAD-related gene expression profiles were screened, including 497 LUAD samples and 54 normal samples. A total of 1598 differentially expressed genes were identified, including 1394 upregulated genes and 204 downregulated genes. The information on biological functions and regulated pathways involved in these differential genes were analyzed by clusterProfiler R package. GO analysis showed that it was mainly involved in the positive regulation of RNA polymerase II transcription, mitotic mitosis, nucleosome assembly, oxygen transport, synaptic transmission, and other biological processes. At the same time, they also participate in the extracellular space, extracellular matrix of proteins, nucleosomes, and other cytological components and participate in some protein binding. KEGG pathway analysis showed that this differentially expressed gene was mainly involved in neural active ligand-receptor interaction, amino acid biosynthesis, calcium ion signaling pathway, PI3K-Akt signaling pathway, etc. The differential gene PPI interaction network was constructed through the String database, combined with the MCC algorithm in Cytohubba plug-in Cytoscape, and 10 key genes were finally identified, namely CCNA2, CDC20, CCNB2, KIF11, TOP2A, BUB1, BUB1B, CENPF, TPX2, and KIF2C. The GEPIA database is a visual big data analysis platform for cancer based on two well-known transcriptome databases, which are TCGA and GTEx. GEPIA database was used to analyze the expression of each gene in normal and cancer cells. Survival and SurvMiner of R package analyzed the influence of each gene on the overall survival rate of LUAD patients and further verified the accuracy of key gene screening.

Cyclin A2 (CCNA2) and cyclin B2 (CCNB2) belong to the cyclin family and are key regulators of a cell cycle [7]. They have been shown to be significantly overexpressed in a variety of cell cycles and are associated with the development and recurrence of lung cancer, breast cancer, colorectal cancer, and other cancers [8–12]. CDC20, a class of proteins encoding periodic kinases, belongs to the cell division cycle gene family. It has been reported that it is likely to be an oncogenic protein, which is overexpressed in a variety of poorly differentiated tumor cells, including lung cancer, colorectal cancer, breast cancer and bladder cancer, and is associated with their poor prognosis [13–16].

KIF11, a kinesin superfamily gene, is a spindle motor protein encoded by kinesin Eg5 gene and involved in the formation of mitotic spindles [17]. Ling et al. found that the overexpression of KIF11 in lung cancer was related to advanced pathological grade and lymph node metastasis, suggesting that KIF11 may be an effective target for lung cancer prevention and treatment [18]. DNA topoisomerase II Alpha (TOP2A) is encoded by TOP2A gene, which controls and changes the topological state of DNA during transcription and is involved in mitosis of various malignant tumor cells. It has been reported that TOP2A overexpression is closely related to the proliferation, invasion, and interference of NSCLC [19]. BUB1 is a serine/threonine protein kinase encoded by the human BUB1 gene, which plays a key role in centromere binding and spindle checkpoint activation during mitosis. Jiang et al. showed that phosphorylation of CDC20 may help BUB1 to achieve effective regulation of cell cycle [20]. BUB1B, an enzyme encoded by BUB1B gene, is significantly overexpressed in lung cancer, bladder cancer, gastric cancer, colon cancer, liver cancer, and other tumors and plays an important role in the occurrence and development of tumors [21]. Centromere Protein F(CENPF) is a key protein in cell cycle regulation. Previous studies have shown that overexpression of CENPF may be closely related to the occurrence, development, and prognosis of prostate cancer, liver cancer, breast cancer, and other malignant tumors, but its effect on LUAD is rarely reported [22]. Targeting Xenopus kinesin-like protein 2 (TPX2), a microtubule-associated protein involved in spindle assembly, plays a vital role in the induction of peripheral assembly and growth in M phase, and is also overexpressed in a variety of human tumors to promote tumorigenesis develop. It has been reported that TPX2 overexpression is associated with a poor prognosis of NSCLC, suggesting that TPX2 may become a prognostic gene [23]. KIF2C, a mitotic centromere-associated kinesin, is involved in microtubule depolymerization and chromosome segregation and regulates mitosis and cell cycle. Abnormal expression of KIF2C can lead to chromosome misalignment in S phase, chromosome misseparation in G2 phase, and stimulate the occurrence and development of tumors [24].

This study provides a basis for the treatment of LUAD, but it lacks validation from relevant in vivo and in vitro experiments, so the next step of work will be to conduct experiments to validate the mechanism of these hub genes with a view to providing new directions for clinical treatment.

## 5. Conclusion

In summary, 10 key genes related to the occurrence, development, and prognosis of LUAD were screened out based on the TCGA database. *CCNA2*, *CDC20*, *CCNB2*, *KIF11*, *TOP2A*, *BUB1*, *BUB1B*, *CENPF*, *TPX2* and *KIF2C* were significantly overexpressed in LUAD as well as plays an important role in the LUAD cell cycle. These results suggest that these genes have great potential in the subsequent prevention, treatment, and prognosis of LUAD, which can provide a certain reference value for the diagnosis and drug treatment of LUAD.

## Figures and Tables

**Figure 1:** Heat map and volcano map of differentially expressed genes. (a) Heat map of the top 50 genes with the most significant differences. (b) Volcano map of differential genes (red dots: significantly upregulated genes, blue dots: significantly downregulated genes, gray dots: genes with no significant differences).

**Figure 2:** GO and KEGG enrichment analysis of differential genes. (a) GO enrichment analysis of 1394 upregulated genes. (b) KEGG enrichment analysis of 1394 upregulated genes. (c) GO enrichment analysis of 204 downregulated genes. (d) KEGG enrichment analysis of 204 downregulated genes.

**Figure 3:** Screening of top 10 hub genes based on PPI network. (a) Top 50 gene-protein interaction network diagram. (b) MCC algorithm was used to screen the top 10 central genes.

**Figure 4:** Expression levels of 10 hub genes in lung adenocarcinoma. (a–j) BUB1, BUB1B, CCNA2, CCNB2, CDC20, CENPF, KIF2C, KIF11, TOP2A, and TPX2 (Red: lung adenocarcinoma tissue, Grey: normal lung tissue.). ∗ represents *P* < 0.05, the difference is significant.

**Figure 5:** Overall survival analysis of 10 hub genes. (a–j) BUB1, BUB1B, CCNA2, CCNB2, CDC20, CENPF, KIF2C, KIF11, TOP2A, and TPX2.

## Data Availability

All data, models, and code generated or used during the study appear in the submitted article.
